# Invasion inhibition in pancreatic cancer using the oral iron chelating agent deferasirox

This article has been retracted.

**DOI:** 10.1186/s12885-020-07167-8

**Published:** 2020-07-22

**Authors:** Shogo Amano, Seiji Kaino, Shuhei Shinoda, Hirofumi Harima, Toshihiko Matsumoto, Koichi Fujisawa, Taro Takami, Naoki Yamamoto, Takahiro Yamasaki, Isao Sakaida

**Affiliations:** 1 Department of Gastroenterology and Hepatology, Yamaguchi University Graduate School of Medicine, 1-1-1 Minami-Kogushi, Ube, Yamaguchi 755-8505 Japan; 2 Department of Oncology and Laboratory Medicine, Yamaguchi University, Graduate School of Medicine, Ube, Yamaguchi Japan

**Keywords:** Pancreatic cancer, Iron chelation, Cancer therapy, Rho family protein, Deferasirox, Invasion

## Abstract

**Background:**

Iron is required for cellular metabolism, and rapidly proliferating cancer cells require more of this essential nutrient. Therefore, iron regulation may well represent a new avenue for cancer therapy. We have reported, through in vitro and in vivo research involving pancreatic cancer cell lines, that the internal-use, next-generation iron chelator deferasirox (DFX) exhibits concentration-dependent tumour-suppressive effects, among other effects. After performing a microarray analysis on the tumour grafts used in that research, we found that DFX may be able to suppress the cellular movement pathways of pancreatic cancer cells. In this study, we conducted in vitro analyses to evaluate the effects of DFX on the invasive and migratory abilities of pancreatic cancer cells.

**Methods:**

We used pancreatic cancer cell lines (BxPC-3, Panc-1, and HPAF II) to examine the efficacy of DFX in preventing invasion in vitro, evaluated using scratch assays and Boyden chamber assays. In an effort to understand the mechanism of action whereby DFX suppresses tumour invasion and migration, we performed G-LISA to examine the activation of Cdc42 and Rac1 which are known for their involvement in cellular movement pathways.

**Results:**

In our scratch assays, we observed that DFX-treated cells had significantly reduced invasive ability compared with that of control cells. Similarly, in our Boyden chamber assays, we observed that DFX-treated cells had significantly reduced migratory ability. After analysis of the Rho family of proteins, we observed a significant reduction in the activation of Cdc42 and Rac1 in DFX-treated cells.

Conclusions: DFX can suppress the motility of cancer cells by reducing Cdc42 and Rac1 activation. Pancreatic cancers often have metastatic lesions, which means that use of DFX will suppress not only tumour proliferation but also tumour invasion, and we expect that this will lead to improved prognoses.

## Background

Patients with pancreatic cancer have exceedingly poor prognoses, and in the United States, the 5-year survival rate of the disease is 6%—a staggeringly low number [1]. In Japan, the condition in nearly half of all pancreatic cancer patients is detected at the metastatic state [2], and the fact that pancreatic cancer often exhibits strong invasive and metastatic tendencies is thought to be one reason for poor patient prognoses [1]. The first-choice therapy for unresectable pancreatic cancer is chemotherapy, and over the last 20 years, gemcitabine (GEM) has come to be used as the primary standard therapy [3]. In recent years, FOLFIRINOX therapy [4], a combination of fluorouracil, irinotecan, oxaliplatin, and leucovorin [4], and GEM plus nab-paclitaxel [5] has been reported to be useful. However, while these kinds of combination chemotherapies have comparatively higher therapeutic effects than GEM monotherapy, they also have higher incidence rates of side effects like cytopenia. Furthermore, more than half of all pancreatic cancer patients are diagnosed at age 65 or older [6]. Consequently, it is vital, especially for elderly pancreatic cancer patients, that new chemotherapies with low side-effect incidence rates be studied.

Iron is required for cellular replication, metabolism, and proliferation [7]. Cancer cells proliferate rapidly, causing them to need more iron than normal cells; thus, iron regulation therapy may represent a new avenue for cancer therapy [8]. Iron chelators are existing drugs that are prescribed for iron overload. Because they are not anticancer drugs, they have very few side effects. We were the first to report the clinical effectiveness of the iron chelator deferoxamine (DFO) on advanced hepatocellular carcinoma refractory to chemotherapy [9]. Because DFO is an intravenously administered drug, the orally administrable, outpatient-suited, next-generation iron chelator deferasirox (DFX) has begun to be used in recent years. Much is still unknown regarding the mechanism of action of iron chelators. We have investigated the ability of DFX ability to suppress tumour proliferation, and found that it suppresses proliferation in a concentration-dependent manner [10], it improves sensitivity to GEM [11], and that the combination of DFX and sorafenib is better than DFX alone at suppressing liver cancer [12]; we have also examined other secondary effects of iron chelators. Upon conducting a supplementary microarray analysis of the in vivo samples used [10], we observed that the expression of Rho-family genes like *Rac1* and *Cdc42*, involved in cellular movement pathways, was altered in DFX-treated cells, and have begun to consider the possibility that DFX could reduce the metastatic and invasive capabilities of cancer cells. Finally, in recent years, it has been reported that, even in stage II and III pancreatic cancer according to the American Joint Committee on Cancer, 8th Edition, cancer cells appear in peripheral blood and are a useful predictive indicator of patient prognosis [13]. Thus, the importance of elucidating the mechanisms of invasion and their prevention and treatment led to the idea of this study. Here, we conducted in vitro analyses to evaluate the effects of DFX on the invasive and migratory abilities of pancreatic cancer cells.

## Methods

### Cell culture

We used the pancreatic cancer cell lines BxPC-3, Panc-1, and HPAF II, purchased from the American Type Culture Collection (Manassas, VA, USA). All of these cell lines are epithelial cells derived from cancer cells. BxPC-3 cells were cultured in RPMI-1640 (Life Technologies, Carlsbad, CA, USA) with 10% foetal calf serum (FBS) and 50 μg/ml gentamicin. Panc-1 cells were cultured in Dulbecco’s modified Eagle’s medium (Life Technologies) with 10% FBS and 50 μg/ml gentamicin. HPAF II cells were cultured in Eagle’s medium (Life Technologies) with 10% FBS and 50 μg/ml gentamicin. Culture was performed in a 37 °C, 5% CO_2_ environment.

### Reagents

The oral iron chelator DFX was obtained from Novartis (Basel, Switzerland). For in vitro studies, DFX was dissolved in dimethyl sulphoxide at a stock concentration of 100 mM and was used at the concentrations indicated in the results and figures by dilution in culture medium containing 10% FBS (172,012; Sigma-Aldrich, St. Louis, MO, USA). For in vivo studies. DFX was dissolved in sodium chloride solution (0.9% w/v; Chemix Inc., Yokohama, Japan).

#### Trypan blue exclusion assay

Cell viability of pancreatic cancer cell lines under treatment with DFX (0, 10, 50, 100 μM) was evaluated. Each pancreatic cancer cell line was cultured in an environment of 37 °C, 5% CO_2_. DFX (0, 10, 50, 100 μM) was added and the cells were incubated for 48 h, after which equal amounts of 0.4% Trypan blue solution (Life Technologies) was added to the cell suspensions, and the viability of each pancreatic cancer cell line was assessed using the Countess Automated Cell Counter (Invitrogen, CA, USA).

### Wound-healing scratch assay

The migratory ability of pancreatic cancer cells was evaluated using a wound-healing assay. Each pancreatic cancer cell line was cultured at 37 °C and 5% CO_2_ in 6-well culture plates (BD Biosciences, San Jose, CA, USA) to 80% confluence. The suspended cells were removed with three washes of phosphate-buffered saline (PBS). A sterilised pipette tip was then used to create a wound (scratch) in the confluent layer. Next, DFX (0, 10, 50, or 100 μM), the Rac-1 inhibitor NSC 23766 (0, 50, 100, 200 μM; Selleck, Houston, TX, USA), or the Cdc42 inhibitor ML141 (0, 10, 20, 40 μM; Selleck) were added to each well, and the cells were incubated for 24 h. Afterwards, the wound width was measured; the ratio of pre- and post-culture wound widths was used as an index of cell migration, and comparisons were made with the control group.

### Boyden chamber assay

To assess invasion ability, we used 24-well Boyden chamber assays (CytoSelect 24-Well Cell Invasion Assay Kits, CELL BIOLABS, San Diego, CA, USA). Each pancreatic cancer cell line was cultured in the upper chamber (at 1.0 × 10^6^ cells/insert), and serum-free medium containing DFX (0, 10, 50, or 100 μM) was added to each chamber. Culture medium with 10% FBS was used in the lower well. Cells were cultured at 37 °C and 5% CO_2_ for 96 h. After 96 h, the cells remaining in the upper chamber were removed, and the chamber was tilted several times in detachment solution to completely detach the cells from the membrane. CyQuant® was added to each well, and after 20 min of incubation at room temperature, a multimode reader (Infinite 200 PRO, Tecan Trading, AG, Switzerland) was used to measure fluorescence at 480 nm/520 nm, which was then compared to that of the control group.

### Rho GTPase activity assay

GTP-bound Rac1 and Cdc42 were measured using corresponding G-LISA Activation Assay Kits (Cytoskeleton, Denver, CO, USA). After stimulation, cells were washed twice with cold PBS and lysed using the lysis buffer provided with the kits for 15 min on ice. The lysates were centrifuged at 10,000×*g* for 1 min at 4 °C. Supernatants were aliquoted, snap-frozen in liquid nitrogen, and stored at − 80 °C according to the manufacturer’s protocol. Protein concentrations were determined, and Rho GTPase activity was assessed according to the manufacturer’s instructions.

### Fluorescent phalloidin (F-actin) staining

DFX (0 or 50 μM) was added to BxPC-3 cells, and they were cultured at 37 °C and 5% CO_2_ for 24 h. The culture medium was removed and cells were washed with PBS. Subsequently, 200 μL of cell fixative (4% formaldehyde in PBS) was added, and cells were left for 10 min at room temperature for fixing. Afterwards, cells were washed with PBS and permeabilisation buffer (0.5% Triton X-100 in PBS) was added and incubated at room temperature for 5 min. Next, 200 μL of 100 nM Acti-stain™ 488 phalloidin (Cytoskeleton, Denver, CO, USA) was added, and after 30 min of dark-room incubation, cells were viewed using a multi-confocal laser microscope (Zeiss, LSM710 system, Oberkochen, Germany).

### Statistical analyses

Analyses performed were the Student’s t test or nonparametric ANOVA test, using the statistical analysis software JMP13 (SAS Institute Inc., Cary, NC, USA). Results are expressed as mean ± standard deviation (SD). *P* values < 0.05 were deemed significant.

## Results

### DFX does not affect the cell viability of pancreatic cancer cells in vitro

We assessed the effect of DFX on the viability of pancreatic cancer cells treated with DFX for 48 h. No obvious decline was seen in the survival rates for treatments with DFX at 10 μM, 50 μM, and 100 μM in all cell lines (BxPC-3, Panc-1, and HPAFII), as compared to the control group (Fig. 1).

**Fig. 1:** Cell viability of pancreatic cancer cell lines treated with DFX. BxPC3, Panc1, and HPAFIIwere treated with DFX (0, 10, 50, or 100 μM) for 48 h and stained with trypan blue to evaluate cell viability (*n* = 3)

### DFX attenuates the migratory and invasive abilities of pancreatic cancer cells in vitro

To evaluate the effect of DFX on pancreatic cancer cell line migration ability, a scratch assay was conducted. In addition, because the results of a micro-array analysis showed a decline in expression of Rac1 and Cdc42, similar experiments were performed with the Rac1 inhibitor NSC 23766 and the Cdc42 inhibitor ML141. A significant decline in migration ability was seen in the DFX 10 μM, 50 μM, and 100 μM treatment groups for BxPC-3, Panc-1, and HPAFII, as compared to the control group (Fig. 2). In addition, compared to the control cells, a significant decline in migration ability was achieved with as low as 50 μM NSC 23766 in BxPC-3 and HPAFII. In Panc-1, 100 μM and 200 μM NSC 23766 caused a significant decline in migration ability (Fig. 3). Similarly, treatment with up to 40 μM ML141 resulted in a significantly declined migration ability in BxPC-3, Panc-1, and HPAFII (Fig. 3). For further evaluation of migration ability in DFX treated pancreatic cancer cell lines, a Boyden chamber assay was conducted. In BxPC-3, HPAFII, and Panc-1, we confirmed a significant abrogation of migration following treatment with DFX at 10 μM, 50 μM, and 100 μM, as compared to the control cells (Fig. 4).

**Fig. 2:** Effect of DFX on migratory ability of pancreatic cancer cells. Pancreatic cancer cell lines (BxPC-3, Panc-1, HPAFII) were treated with DFX (0, 10, 50, 100 μM) and incubated for 24 h. **a**-**c** Migrated cells were visualized via phase-contrast microscopy. **d**-**f** % wound closure was measured and the ratio to wound width at the start of the incubation was used as an index of cell migration, compared to control group (*n* = 3 each). Data are presented as mean ± SD. *P < 0.01 vs control

**Fig. 3:** Effect of NSC 23766 and ML141 on the invasion ability of pancreatic cancer cells. Pancreatic cancer cell lines (BxPC-3, Panc-1, HPAFII) were treated with either NSC 23766 (0, 50, 100, 200 μM) or ML141 (0, 10, 20, 40 μM), and incubated for 24 h. **a**-**c**, **g**-**i** Migrated cells were visualised via phase-contrast microscopy. **d**-**f**, **j**-**l** % wound closure was measured, and the ratio to wound width at the start of the culture was used as an index of cell migration to conduct a comparative evaluation against the control group (*n* = 3). Data are presented as mean ± SD. *P < 0.05, **P < 0.01 vs control

**Fig. 4:** Effect of DFX on invasive ability of pancreatic cancer cells. **a**–**c** Pancreatic cancer cells were cultured in the upper chamber, and serum-free medium containing DFX (0, 10, 50, or 100 μM) was added to each chamber. After 96 h of incubation, a multimode reader was used to measure fluorescence at 480 nm/520 nm, which was then compared to that of the control group (*n* = 3). Data are presented as mean ± SD. *P < 0.05

### DFX reduces activation of rho family proteins Rac1 and Cdc42 in vitro

To assess the contributions of Rho/Rac1/Cdc42 signaling in DFX-suppressed cell migration, we analysed the expression of Rho family proteins in DFX-treated pancreatic cancer cell lines using G-LISA. We observed a significant decline in Rac1 expression in BxPC-3 cells treated with 50 μM and 100 μM DFX, as compared to the control group. In addition, in Panc-1, a significant decline in Rac1 expression was seen in the DFX 100 μM treatment group. The HPAFII cells also showed a trend toward reduced expression of Rac1 in the DFX groups as compared to the control group, though this difference was not significant (Fig. 5). Assessment of Cdc42 levels showed a significantly declined expression in the BxPC-3 cells treated with DFX at 50 μM and 100 μM, as compared to the control group. Panc-1 and HPAFII cells also showed a significant decline in Cdc42 expression in the DFX 10 μM, 50 μM and 100 μM treatment groups, as compared to the control group (Fig. 6). Phalloidin staining was also performed on BxPC3 cells treated with DFX, revealing a significant reduction in filopodia in the DFX treatment group, compared with the control cells (Fig. 7).

**Fig. 5:** Effect of DFX on Rac1 activation in pancreatic cancer cells. Pancreatic cancer cells were treated with DFX (0, 10, 50, or 100 μM); after 48 h of incubation, Rac1 activation was measured using G-LISA in (**a**) BxPC-3 cells(*n* = 3), **b** Panc-1 cells (*n* = 3), and (**c**) HPAF II cells (*n* = 3). Data are presented as mean ± SD. *P < 0.05, **P < 0.01

**Fig. 6:** Effect of DFX on Cdc42 activation in pancreatic cancer cells. Pancreatic cancer cells were treated with DFX (0, 10, 50, or 100 μM); after 48 h of incubation, Cdc42 activation was measured using G-LISA in (**a**) BxPC-3 cells (*n* = 3), **b** Panc-1 cells (*n* = 3), and **c** HPAF II cells (*n* = 3). Data are presented as mean ± SD. *P < 0.05, **P < 0.01

**Fig. 7:** BxPC-3 cells stained with phalloidin-rhodamine. DFX (0, 50 μM) was added to BxPC-3 cells and incubated for 24 h. Phalloidin staining was performed and cells observed with a multi-confocal microscope to measure the number of filopodia (*n* = 13). Scale bars indicate 50 μm. Data are presented as mean ± SD. *P < 0.01

## Discussion

The effectiveness of iron chelators on cancer was first reported in leukaemia in 1986 [14, 15], and since then, the effectiveness of DFX on a variety of carcinomas has been reported [9, 10, 16–19]. Furthermore, in recent years, reports [20, 21] have indicated that administration of iron chelators in prostate and colon cancer inhibits TGF-β and promotes the expression of N-myc downstream regulated gene-1, a metastasis suppression factor, to suppress cell invasion. However, the mechanisms by which these effects are achieved is still poorly understood.

Rac1 and Cdc42 are Rho-family G proteins that have been linked to a variety of different cancers and are involved in epithelial to mesenchymal transition, cell-cycle progression, migration/invasion, tumour growth, angiogenesis, and oncogenic transformation. Rac1 and Cdc42 are generally overexpressed or overactivated in cancer cells [22]. In Rho-family G proteins, guanine nucleotide exchange factors work to allow GDP-GTP exchange and activate the protein. In contrast, GTPase-activating protein promotes GTP hydrolysis to inactivate these proteins [23]. Rac1 and Cdc42 are important signal transduction molecules whose dysregulation is associated with cancer occurrence and cell migration/invasion [24]. Reports have shown that in cases of pancreatic cancer, highly elevated expression of Cdc42 is significantly correlated with poor prognosis [25]. It has been predicted that suppressing the activity of Rac1 and Cdc42 will reduce invasive capability.

This study was an in vitro analysis to evaluate the effect of the iron chelator DFX, on the migration/invasion of pancreatic cancer cell lines. Our previous paper showed an elevated caspase-3 activity at 48 h after treatment with 50 or 100 μM DFX [10]. Induction of apoptosis by DFX treatment may thus have contributed to suppress migration/invasion, though we confirmed the higher cellular viability of pancreatic cancer cells at 48 h after DFX treatment (Fig. 1). Our results also suggested that DFX may not only demonstrate the tumor growth inhibitory effect that we reported previously, but may also reduce the migration/invasion of pancreatic cancer cells by abrogating the expression of invasion-related Rho-family G proteins, Rac1 and Cdc42. Previous studies have reported that iron chelator treatment suppresses ROCK expression with consequent reduction of actin polymerization [20], and suppression of N-cadherin expression that resulted in blocking the invasiveness of esophageal cancer cells [26]. However, this is the first study to report the changes caused by iron chelators in cell shape and in reducing migration ability through suppression of Rac1 and Cdc42.

Rac1 and Cdc42 may well be valid and effective therapeutic targets in the treatment of cancer. The literature shows that administration of Rac1 and Cdc42 inhibitors suppresses migration and invasion in breast cancer models [27]. Additionally, reports indicate that inhibition of Rac1 increases the susceptibility of pancreatic and breast cancers to radiation therapy [28, 29]. In any case, many studies are being performed on these compounds and their links with cancer.

The strong invasive tendency of pancreatic cancer is a factor that leads to its poor prognosis [1]; thus, suppressing Rac1 or Cdc42 and thereby controlling invasion may be clinically effective. For example, at present, as recommended by the National Comprehensive Cancer Network guidelines, preoperative adjuvant therapies are actively performed in resectable, border region (BR) pancreatic cancers [30]. However, almost no evidence recommends a specific preoperative adjuvant therapy regimen for BR cases. While FOLFIRINOX or GEM + albumin-bound paclitaxel therapies are the most approved [31, 32], the addition of an iron chelator like DFX would contribute the tumour-proliferation-suppressive effects of this class of drug as well as its suppressive effects on the emergence of metastatic lesions during chemotherapy treatment, owing to the iron chelator’s ability to reduce Rac1 and Cdc42 activation. Furthermore, because iron chelators are known medications that are commonly used to treat iron overload, the fact that they are not anticancer drugs means that their addition to anticancer drug regimens should cause little to no adverse effects; this is another advantage of this class of therapies. However, because this study was an in vitro analysis, future evaluations of protein expression changes and invasive ability in vivo or in human pancreatic cancer should lead to a more thorough understanding.

## Conclusions

In this study, after administration of DFX to pancreatic cancer cell lines, we confirmed significant reductions in the activation of Rac1 and Cdc42. In scratch assays and Boyden chamber assays, we also observed significant reductions in cell migratory and invasive abilities. This is the first paper to report that DFX has the ability to suppress tumour proliferation (as we have previously reported), as well as to reduce the abilities of pancreatic cancer cells to change shape and migrate by reducing the activation of Rac1 and Cdc42, Rho-family G proteins involved in cancer invasion.

## Data Availability

The microarray data have been deposited in the NCBI’s Gene Expression Omnibus (GEO) under GEO series accession no. GSE81363 [10]. The other datasets used and/or analysed during the current study are available from the corresponding author on reasonable request.

## Abbreviations

GEM: Gemcitabine
DFO: Deferoxamine
DFX: Deferasirox
FBS: Foetal calf serum
PBS: Phosphate-buffered saline
SD: Standard deviation
BR: Border region
